# Accuracy of Focused Assessment with Sonography for Trauma (FAST) in Blunt Abdominal Trauma

**DOI:** 10.1155/2022/8290339

**Published:** 2022-10-07

**Authors:** Tae Ah Kim, Junsik Kwon, Byung Hee Kang

**Affiliations:** ^1^Division of Hepatobiliary and Pancreatic Surgery, Department of Surgery, Ulsan University College of Medicine and Asan Medical Center, Seoul, Republic of Korea; ^2^Division of Trauma Surgery, Department of Surgery, Ajou University School of Medicine, Suwon, Republic of Korea

## Abstract

**Purpose:**

This study aimed to evaluate the accuracy and outcomes of focused assessment with sonography for trauma (FAST) and determine the factors associated with true-positive FAST results.

**Methods:**

The FAST results from 2016 to 2020 were retrospectively reviewed. Cases involving penetrating injury, transfer from other hospitals, age ≤ 16 years, prehospital arrest, and no confirmatory test were excluded. Intra-abdominal fluid was confirmed using computed tomography or operative findings. The sensitivity, specificity, positive predictive value (PPV), and negative predictive value (NPV) were calculated. Demographic data, injury characteristics, and outcomes were compared between true-positive and false-negative results. Logistic regression was used to identify the factors associated with true-positive results.

**Results:**

Of 2,758 patients, 163 and 2,595 patients showed positive and negative results, respectively. True positives were 135 and true negatives were 2325. The overall sensitivity, specificity, PPV, and NPV were 33.3%, 98.8%, 82.8%, and 89.6%, respectively. The sensitivity increased to 49.1% in patients with initial systolic blood pressure (SBP) ≤ 90 mmHg. The true-positive group showed a lower SBP and Glasgow Coma Scale score and a higher laparotomy rate than the false-negative group. However, mortality showed no significant difference. In logistic regression analysis, hollow viscus injury (1.820 [1.123–2.949], *P*=0.015) and the lowest SBP (0.988 [0.980–0.997], *P*=0.009) were associated with true-positive results compared to false-negative results.

**Conclusion:**

The overall sensitivity of FAST was low; therefore, it should be performed in selected patients such as SBP ≤ 90 mmHg. Because of its low sensitivity and no influence on outcome, physicians should not rely solely on FAST.

## 1. Introduction

Focused assessment with sonography for trauma (FAST) is a rapid and useful diagnostic method for detecting free fluid in trauma patients [1]. FAST continues to gain popularity since it is easy to learn, readily accessible, and portable, and its coverage extends to the thorax [2]. FAST is the world's widely accepted procedure in trauma care, and about 68% of physicians working at emergency medical centers use FAST as one of point-of-care ultrasonography in the Republic of Korea [3]. Moreover, residents of the general surgery and emergency department should learn FAST during training, and FAST seems to be gaining popularity in this regard.

Despite its advantages, the accuracy of FAST is variable. The sensitivity, specificity, positive predictive value (PPV), and negative predictive value (NPV) have been reported to be in the range from 28–76%, 83–97%, 87–96%, and 37–94%, respectively [4–9]. However, no previous studies have evaluated the accuracy of FAST in the Republic of Korea except for few experimental studies and those conducted by emergency medical technicians [10, 11]. In addition, FAST may show false-negative results because of its low sensitivity, and the influence of false-negative FAST results on patient outcomes is inconclusive. Thus, the purpose of this study was to survey the accuracy of FAST and estimate the association between false-negative FAST results and outcomes.

## 2. Methods

The findings for patients who underwent FAST in the trauma bay of the trauma center from January 2016 to December 2020 were retrospectively reviewed. More than 1,500 injured patients are admitted to the trauma bay of our trauma center annually, and trauma surgeons usually perform FAST. The trauma center has two entrances for injured patients: prehospital triage performed by emergency medicine personnel for major trauma patients to the trauma bay and minor trauma patients to the emergency room. Therefore, FAST is routinely performed in patients with blunt trauma with a high-risk injury mechanism. In our protocol, computed tomography (CT) could be performed more readily because of the possibility of abdominal injury and relatively cheap cost of CT owing to the national health insurance system. The exclusion criteria were as follows: prehospital arrest, penetrating trauma, transfer from another hospital, age ≤16 years, and no further evaluation such as CT or laparotomy. Intra-abdominal free fluid was confirmed using CT or operative findings. However, in this study, the fluid amount was not considered.

The sensitivity, specificity, PPV, and NPV of the FAST results were calculated, and a subgroup analysis based on blood pressure was carried out. Patients were dichotomized into true-positive and false-negative groups, and their demographic data, vital signs, injury characteristics, treatment, and outcomes were compared. The abdominal injury site was categorized based on the abbreviated injury scale (AIS), and gastrointestinal injuries were combined with hollow viscus injuries. Abdominal organ injury was defined by an AIS score ≥3, which usually requires surgery. The logistic regression analysis excluded retroperitoneal organ (the kidneys and pancreas) injuries as they may not produce intra-abdominal fluid.

Continuous variables were presented as the mean ± standard deviation, and categorical variables were presented as the number (percentile). Student's *t*-test or the Mann–Whitney test was utilized for analysis of continuous variables, while the chi-square test was performed for categorical variables. After univariate analysis, variables with *P* < 0.05 were included in the multivariate analysis by applying binary logistic regression. All analyses were performed using IBM SPSS version 21.0 (IBM Corp., Armonk, NY, USA). This study was approved by the institutional review board of our institution (AJIRB-MED-MDB-22-038).

## 3. Results

Of 4,484 patients, 2,758 patients, including 163 and 2,595 patients showing positive and negative FAST results, respectively, were selected after applying the exclusion criteria. A total of 405 (14.7%) patients had intra-abdominal free fluid (Figure 1).

The overall sensitivity, specificity, PPV, and NPV of FAST were 33.3%, 98.8%, 82.8%, and 89.6%, respectively. However, in patients with initial systolic blood pressure (SBP) ≤ 90 mmHg or lowest SBP during resuscitation in the trauma bay ≤90 mmHg, sensitivity increased to 49.1% and 48.3%, respectively (Table 1).

The true-positive and false-negative FAST groups included 135 and 270 patients, respectively. The true-positive group had a lower SBP and Glasgow Coma Scale score and more transfusions. Moreover, laparotomy cases were more frequent in the true-positive group than in the false-positive group, but no significant difference was noted in mortality and intensive care unit length of stay (Table 2).

Hollow viscus, pancreas, and vascular injuries were more frequent in the true-positive group than in the false-negative group; however, kidney injury was more frequent in the false-negative group. Other solid organ injuries were not significantly different between the two groups (Table 3).

In multivariate analysis, the lowest SBP (0.988 [0.980–0.997], *P*=0.009) and hollow viscus injury (1.820 [1.123–2.949], *P*=0.015) were associated with true-positive FAST results in patients with intra-abdominal free fluid (Table 4).

## 4. Discussion

In this study, the overall sensitivity of FAST was 33.3% and the number of false-negative cases was larger than that of true-positive cases. The sensitivity of FAST was lower than that reported in other studies (43–76%) [3–6, 9]. Branney et al. reported that the mean volume of fluid detected in ultrasonography at Morrison's pouch was 619 mL, and only 10% of the cases showed free fluid less than 400 mL [12]. In this study, intra-abdominal free fluid was defined based on CT or operative findings; however, the amount of fluid was not considered. Therefore, some patients with minimal hemoperitoneum may have been considered to be showing intra-abdominal free fluid, and these cases could not be distinguished easily. Moreover, only 34.4% of the false-negative cases required laparotomy; thus, the amount of hemoperitoneum may have been small in the false-negative group. Subcutaneous emphysema, bowel gas, and obesity are common obstacles to complete FAST visualization [13]. Additionally, the examiner still had to classify each case as positive or negative despite the inappropriate view because there was no “indeterminate” category. Moreover, although trauma surgeons usually directly perform FAST exams in the trauma bay, there was no official education program for the FAST examination in our center.

Because 85.3% of patients showed no or minor abdominal injury (true-negative or false-positive cases), the value of FAST examinations in cases of blunt trauma with a high-risk injury mechanism is questionable. Natarajan et al. reported that the sensitivity of FAST in the stable group was 41%, which is not worthwhile because of the need for a confirmatory evaluation in such cases [7]. Carter et al. demonstrated that the sensitivity of FAST exams was 21% and 28% in the stable and unstable groups, respectively; thus, the decision to perform laparotomy should not be influenced by a negative FAST result [14]. In the current study, sensitivity and PPV increased when the FAST examination was performed in patients with initial SBP ≤ 90 mmHg or lowest SBP ≤ 90 mmHg. For hemodynamically stable patients, the FAST examination is not a decision-making procedure because CT is performed for confirmation. Instead, the FAST examination is more helpful for assessment of unstable patients as a rapid, noninvasive bedside procedure. However, it still shows a low sensitivity of approximately 48% in such cases. Thus, the decision to perform exploratory laparotomy should not rely solely on negative FAST results.

A systematic review could not clarify whether FAST-based decisions resulted in better outcomes for blunt abdominal trauma [15]. In this study, false-negative FAST results did not affect the mortality rate and mortality was not significantly different even in initial SBP ≤ 90 mmHg or lowest SBP ≤ 90 mmHg groups. The decision to perform laparotomy was more frequent in the true-positive group; nevertheless, 34.4% of the patients required laparotomy in the false-negative group. In addition to its low sensitivity, FAST is a screening exam and not a definite diagnostic method. Therefore, although a positive FAST result indicates laparotomy, the need for it should not be ruled out in negative FAST results.

Laselle et al. demonstrated that spleen, liver, and vascular injuries were associated with a true-positive FAST result [16]. Carter et al. demonstrated that the spleen was an independent predictor of a positive FAST result [14]. In contrast, hollow viscus injury was associated with a true-positive FAST exam in the current study. Unlike other studies that used the International Classification of Disease codes, this study used the AIS codes. Generally, bowel injury is not detectable in FAST examinations. However, AIS coding classifies mesentery injury without a named vessel as an internal organ injury; therefore, mesentery bleeding was classified under hollow viscus. In addition, we included only organ injury cases with AIS ≥3, and minor lacerations in solid organs that could cause hemoperitoneum were excluded. Schnuriger et al. reported that the false-negative rate of FAST was about 20–44% in grade I–II solid organ (liver or spleen) injury, but it was 0–12% in grade III–V injury [17]. Thus, the results could be different if all injuries were included. Nevertheless, unlike grade III solid organ injury, grade III hollow viscus injury usually requires surgery; therefore, surgeons should consider laparotomy in FAST-positive cases.

This study had several limitations. First, the patients in the true intraperitoneal fluid group included those with physiologic intra-abdominal fluid or a small amount of fluid collection. However, FAST indicates intra-abdominal fluid regardless of the need for treatment, and it cannot distinguish cases with a clinically meaningful amount of fluid. Second, the findings did not reflect the results of repeated FAST examinations. In the current study, if the FAST result changed from negative to positive, the exam was reported to be positive. In such cases, the timing of the exam may have affected the results, but this factor was not considered. Third, false-positive FAST results could also complicate the decision to perform laparotomy. However, the number of false-positive FAST results was too small for analysis, and further studies are needed in this regard.

In conclusion, FAST showed low sensitivity and more false-negative cases than true-positive cases. To increase its sensitivity, FAST should be performed in selected patients, such as those with shock. Laparotomy should be considered in positive FAST cases. However, considering the high number of false-negative cases, surgeons should not rely solely on negative FAST results to make decisions regarding laparotomy.

## Figures and Tables

**Figure 1:** Study population.

**Table 1:** Accuracy of FAST examination according to SBP.

	Sensitivity (%)	Specificity (%)	PPV (%)	NPV (%)
Total	33.3	98.8	82.8	89.6
Initial SBP ≤ 90 mmHg	49.1	96.9	93.1	69.2
Lowest SBP ≤ 90 mmHg	48.3	99.0	95.8	80.2

SBP: systolic blood pressure; PPV: positive predictive value; NPV: negative predictive value. The lowest SBP was defined during initial resuscitation in the trauma bay.

**Table 2:** Patients' characteristics and outcomes.

	True-positive (*n* = 135)	False-negative (*n* = 270)	*P*
Age (years)	45.2 ± 15.7	46.0 ± 17.3	0.654
Sex (male, %)	111(82.2%)	213 (78.9%)	0.598
Body mass index (kg/m^2^)	24.7 ± 4.3	24.8 ± 4.2	0.704^*∗*^
Prehospital time (min)	47.9 ± 21.3	61.9 ± 125.4	0.198

Vital signs			
Initial SBP (mmHg)	117.8 ± 28.7	125.2 ± 27.5	0.008
Lowest SBP (mmHg)	82.2 ± 29.5	94.6 ± 28.9	<0.001
Initial heart rate (/min)	102.5 ± 25.4	97.2 ± 24.1	0.058
Initial respiratory rate (/min)	23.1 ± 6.7	23.4 ± 6.6	0.593

Glasgow Coma Scale	10.8 ± 5.2	11.8 ± 4.5	0.034^*∗*^
Injury severity score	31.3 ± 13.4	28.8 ± 11.8	0.040^*∗*^
Injury mechanism, *n* (%)			0.583
Motor vehicle crash	60 (44.4%)	79 (29.3%)	
Auto versus pedestrian	22 (16.3%)	49 (18.1%)	
Motorcycle	19 (14.1%)	56 (20.7%)	
Bicycle	2 (1.5%)	1 (0.4%)	
Fall	26 (19.3%)	70 (25.9%)	
Assault	5 (3.7%)	11 (4.1%)	
Machine	1 (0.7%)	2 (0.7%)	
Other	0	2 (0.7%)	

Transfusion within 24 h			
Packed red blood cells (U)	12.4 ± 15.4	7.1 ± 10.6	<0.001
Fresh frozen plasma (U)	10.7 ± 14.2	6.3 ± 9.6	0.001

Treatment			
Laparotomy, *n* (%)	88 (65.2%)	93 (34.4%)	<0.001
ICU LOS (days)	9.7 ± 14.0	9.8 ± 18.2	0.957
Hospital LOS (days)	27.6 ± 25.8	26.5 ± 30.5	0.720
Mortality, *n* (%)			

Total	27 (20.0%)	40 (14.8%)	0.186
Initial SBP ≤ 90 mmHg	11 (34.4%) (*n* = 32)	13 (33.3%) (*n* = 39)	0.926
Lowest SBP ≤ 90 mmHg	24 (28.2%) (*n* = 85)	29 (25.2%) (*n* = 115)	0.633

SBP: systolic blood pressure; ICU: intensive care unit; LOS: length of stay. The lowest SBP was defined during initial resuscitation in the trauma bay. ^*∗*^Mann–Whitney test was utilized.

**Table 3:** Injured organs according to the abbreviated injury scale ≥3 in the abdomen.

	True-positive (*n* = 135)	False-negative (*n* = 270)	*P*
Spleen	36 (26.7%)	66 (24.4%)	0.627
Liver	61 (45.2%)	106 (39.3%)	0.253
Kidney	10 (7.4%)	48 (17.8%)	0.005
Hollow viscus	46 (34.1%)	59 (21.9%)	0.008
Pancreas	8 (5.9%)	3 (1.1%)	0.008
Vasculature	16 (11.9%)	15 (5.6%)	0.025
Bladder	6 (4.4%)	5 (1.9%)	0.191

**Table 4:** Univariate and multivariate analyses of factors associated with true-positive results.

	Univariate analysis		Multivariate analysis	
	OR [95% CI]	*P*	OR [95% CI]	*P*
Age	0.997 [0.985–1.010]	0.653	0.996 [0.983–1.009]	0.517
Sex	1.151 [0.681–1.945]	0.598	1.137 [0.660–1.960]	0.643
Initial SBP	0.990 [0.983–0.998]	0.008	0.998 [0.990–1.007]	0.664
Lowest SBP	0.985 [0.978–0.993]	<0.001	0.988 [0.980–0.997]	0.009
Initial heart rate	1.008 [1.000–1.016]	0.059	1.005 [0.996–1.014]	0.272
Vascular injury	2.286 [1.094–4.778]	0.028	1.665 [0.767–3.615]	0.197
Hollow viscus injury	1.848 [1.169–2.923]	0.009	1.820 [1.123–2.949]	0.015

OR: Odds ratio; CI: confidence interval; SBP: systolic blood pressure. Hosmer–Lemeshow goodness of fit (DF = 8), chi-square = 6.916, *P*=0.546.

## Data Availability

No data were used to support this study.
